The article "Identification of Peptides as Novel Inhibitors to Target IFN-γ, IL-3, and TNF-α in Systemic Lupus Erythematosus" was retracted in 2024. Reasons: signs of a paper mill; suspected computer-generated content; unreliable results or conclusions; concerns about the data.

# Identification of Peptides as Novel Inhibitors to Target IFN-*γ*, IL-3, and TNF-*α* in Systemic Lupus Erythematosus

**DOI:** 10.1155/2021/1124055

**Published:** 2021-11-13

**Authors:** Ghulam Mustafa, Hafiza Salaha Mahrosh, Mahwish Salman, Sumaira Sharif, Raheela Jabeen, Tanveer Majeed, Hafsah Tahir

**Affiliations:** ^1^Department of Biochemistry, Government College University, Faisalabad, 38000, Pakistan; ^2^Institute of Molecular Biology and Biotechnology, The University of Lahore, Pakistan; ^3^Department of Biochemistry and Biotechnology, The Women University Multan, Pakistan; ^4^Department of Biotechnology, Kinnaird College for Women, Lahore, Pakistan; ^5^Department of Environmental Sciences, Quaid-i-Azam University, Islamabad, Pakistan

## Abstract

Autoimmune disorder is a chronic immune imbalance which is developed through a series of pathways. The defect in B cells, T cells, and lack of self-tolerance has been greatly associated with the onset of many types of autoimmune complications including rheumatoid arthritis, systemic lupus erythematosus (SLE), multiple sclerosis, and chronic inflammatory demyelinating polyneuropathy. The SLE is an autoimmune disease with a common type of lupus that causes tissue and organ damage due to the wide spread of inflammation. In the current study, twenty anti-inflammatory peptides derived from plant and animal sources were docked as ligands or peptides counter to proinflammatory cytokines. Interferon gamma (IFN-*γ*), interleukin 3 (IL-3), and tumor necrosis factor alpha (TNF-*α*) were targeted in this study as these are involved in the pathogenesis of SLE in many clinical studies. Two docking approaches (i.e., protein-ligand docking and peptide-protein docking) were employed in this study using Molecular Operating Environment (MOE) software and HADDOCK web server, respectively. Amongst docked twenty peptides, the peptide DEDTQAMMPFR with *S*-score of -11.3018 and HADDOCK score of −10.3 ± 2.5 kcal/mol showed the best binding interactions and energy validation with active amino acids of IFN-*γ* protein in both docking approaches. Depending upon these results, this peptide could be used as a potential drug candidate to target IFN-*γ*, IL-3, and TNF-*α* proteins to control inflammatory events. Other peptides (i.e., QEPQESQQ and FRDEHKK) also revealed good binding affinity with IFN-*γ* with *S*-scores of -10.98 and -10.55, respectively. Similarly, the peptides KHDRGDEF, FRDEHKK, and QEPQESQQ showed best binding interactions with IL-3 with *S*-scores of -8.81, -8.64, and -8.17, respectively.

## 1. Introduction

The innate and adaptive immune system controls the defense organization mediated by multiple components and molecules in an organism [1]. Different organs, signaling pathways, and compounds collectively perform various tasks to protect the organism from external and internal damage. Autoimmunity or production of autoantigens mainly brings disaster to the immune system due to inadequate immune tolerance [2]. The defect in the synergistic relationship between innate immunity and adaptive immunity causes severe consequences including autoimmune disorders, inflammations like systemic lupus erythematosus, rheumatoid arthritis, Alzheimer's disease, multiple sclerosis, and many other complications [3].

The article "Identification of Peptides as Novel Inhibitors to Target IFN-γ, IL-3, and TNF-α in Systemic Lupus Erythematosus" was retracted in 2024. Reasons: signs of a paper mill; suspected computer-generated content; unreliable results or conclusions; concerns about the data.

Systemic lupus erythematosus (SLE) is the most common chronic autoimmune inflammatory disorder characterized by the presence of autoantibodies directed against own cells or tissues of the body. It is intermediated by B cells which generate autoantibodies against nuclear antigens, a type III hypersensitivity reaction that causes chronic systemic inflammation and tissue damage in the joints, skin, brain, lungs, kidneys, and blood vessels [4]. The incidence of SLE prevalence has been predominantly recorded in young middle-aged females. According to studies, the highest prevalence can be seen in certain ethnicities, reflected in prevalence rates of approx. 40/100,000 persons in Northern European cohorts with comparison rates of 200/100,000 patients of African-American descent [5]. SLE is multifactorial in its origin with a wide range of clinical and serological manifestations. There have been many efforts to elucidate the pathogenesis of SLE with current recognition of genetic susceptibility, environmental triggers, and disruption in both the innate and adaptive immune systems [6].

Adaptive immunity is an antigen-specific host defense that comprises of B and T lymphocytes and immunoglobulins. The defected immunity in SLE results in a myriad of complications such as decreased T cell signaling, stimulation of autoaggressive T effector cells, and production of autoantibodies. Apart from all these, any dysregulation in B cells that produces proinflammatory cytokines (i.e., IL-1, IL-3, IL-6, IL-23, and TNF-*α*) pushes the inflammatory events and drives the SLE disease. Thus, targeting these B and T cells could be proved as a therapeutic advantage to control SLE [7].

The role of cytokines regarding SLE has collected much interest of scientists. Type I interferon family along with many other cytokines such as interleukins (IL-3, IL-6, IL-10, and IL-17) and tumor necrosis factor (TNF) is seen to be involved in SLE. These interleukins play a significant role in diseases which are linked to inflammation and autoimmunity [4]. This disease has several variants which are genetically linked with pathogenic mechanisms. Genetics and epigenetics are the factors which contribute directly to cause alterations in the cells of both innate and adaptive immune responses [8].

The article "Identification of Peptides as Novel Inhibitors to Target IFN-γ, IL-3, and TNF-α in Systemic Lupus Erythematosus" was retracted in 2024. Reasons: signs of a paper mill; suspected computer-generated content; unreliable results or conclusions; concerns about the data.

Greater than 95% of SLE patients have detectable serum antinuclear antibody (ANA). Anti-ds-DNA antibodies are highly specific for SLE and present in 65–70% of the patients (versus 0.5% of the healthy population). Anti-ds-DNA antibodies, anti-Ro, anti-La, anti-C1q, and anti-Sm antibodies have been demonstrated histologically in renal biopsy specimens. A number of specific antibodies have been associated with a particular expression of SLE. Anti-Ro and antinucleosome antibodies are most strongly linked with cutaneous lupus [9]. Many combination drug therapies have been in practice for the control of clinical manifestations of SLE, but these have been recorded with severe side effects, and also, the patients of SLE still show a higher standardized mortality rate (i.e., of 4.6-fold) with respect to the general population [10]. Therefore, the current study was planned to reveal anti-inflammatory peptides from plant and animal sources using molecular docking approach. The study includes protein-ligand and peptide-protein docking of twenty anti-inflammatory peptides counter to IFN-*γ*, IL-3, and TNF-*α* receptor proteins as targets for the treatment of SLE. In the current study, we have investigated the potential of these peptides as drug candidates to attenuate the inflammatory response and tissue destruction due to activation of proinflammatory cytokines, B cells, and T cells which lead towards autoantibody production.

## 2. Materials and Methods

The study includes the protein-ligand and peptide-protein docking of twenty anti-inflammatory bioactive peptides against three main receptor proteins (i.e., IL-3, TNF-*α*, and IFN-*γ*) that play leading roles in the pathogenesis of SLE. Molecular Operating Environment v.2015.10 (Chemical Computing Group ULC, Montreal, QC, Canada) [11] was employed for ligand-based docking, and HADDOCK v.2.4 [12] an online server was used for peptide-protein docking.

### 2.1. Ligand Database Preparation

An extensive literature survey was performed to explore plant and animal derived bioactive anti-inflammatory peptides. The chemical structures of these ligands were prepared using ACD ChemSketch v.C40E41 (Advanced Chemistry Development, Inc., Toronto, Ontario, Canada) [13] and saved in MOL format in MOE database as ready-to-dock compounds after energy minimization.

### 2.2. Refinement of Receptor Proteins

The three-dimensional structures of IL-3 (PDB ID: 5UV8), IFN-*γ* (PDB ID: 6E3K), and TNF-*α* (PDB ID: 6OP0) were retrieved from protein data bank (https://www.rcsb.org/). Removal of solvent, addition of hydrogen atoms, energy minimization, and 3D protonation were performed using MOE with default parameters, and the minimized structure of each protein was saved to use as receptor protein for docking studies.

The article "Identification of Peptides as Novel Inhibitors to Target IFN-γ, IL-3, and TNF-α in Systemic Lupus Erythematosus" was retracted in 2024. Reasons: signs of a paper mill; suspected computer-generated content; unreliable results or conclusions; concerns about the data.

### 2.3. Ligand-Protein Docking

The active binding pocket of each receptor protein was selected using the site finder tool of MOE. The prepared ready-to-dock library of twenty anti-inflammatory peptides was docked counter to IL-3, IFN-*γ*, and TNF-*α*, and the top three ligands from each protein-ligand docking were selected on the basis of their interactions and *S*-scores. The algorithm of MOE provides top conformations on the basis of binding patterns of ligands with active amino acids of the receptor protein, minimum energy structure, and maximum occupancy of the binding pocket.

### 2.4. Peptide-Protein Docking

IL-3, IFN-*γ*, and TNF-*α* have been extensively studied due to their roles in the pathophysiology of many autoimmune disorders. The dysfunctioning of the signaling pathways of B and T cells leads towards the production of autoantibodies against the body's own tissues and cells. In the literature, many anti-inflammatory compounds have been reported for autoimmune disease; however, in this study, for the first time, peptide-protein docking was employed to explore the inhibitory effects of peptides counter to selected receptor proteins for the treatment of SLE. The most reported twenty anti-inflammatory peptides were used for docking studies against receptor proteins. For peptide-protein docking, the top peptides against each receptor protein were selected, which were obtained from the results of protein-ligand docking and used for further analysis of peptide-protein docking. The sequences of these peptides were retrieved from the literature and subjected to BLASTp to find their homologs. To predict three-dimensional (3D) structure of each peptide, the PDB database was used during BLAST analyses to find the best templates of each peptide using the homology modeling approach. Modeller v.9.21 (Ben Webb, UCSF, CA, USA) [14] was used to predict 3D structures of selected peptides (i.e., DEDTQAMMPFR and KHDRGDEF).

HADDOCK v.2.4 was used to carry out the docking analysis between the best selected peptides and selected target proteins. Educational version of PYMOL Molecular Graphics System v2.0 (Schrödinger, LLC) was used to visualize the docked complexes and draw figures [15].

#### 2.4.1. Molecular Dynamic Simulation

For 120 nanoseconds, Desmond (Schrödinger LLC) was used to model molecular dynamics in triplicates [16]. The earliest phase of protein-ligand complex for molecular dynamics simulation was used in the docking experiments. Molecular docking studies can predict ligand binding state in static situations. Docking is useful because it provides a static view of a molecule's binding pose at the active site of a protein [17]. By integrating Newton's classical equation of motion, MD simulations typically compute atom movements over time. Simulations were used to predict the ligand binding status in the physiological environment [18, 19].

The article "Identification of Peptides as Novel Inhibitors to Target IFN-γ, IL-3, and TNF-α in Systemic Lupus Erythematosus" was retracted in 2024. Reasons: signs of a paper mill; suspected computer-generated content; unreliable results or conclusions; concerns about the data.

The protein–ligand complex was preprocessed using Protein Preparation Wizard or Maestro, which included complex optimization and minimization. All of the systems were prepared using the System Builder tool. TIP3P (transferable intermolecular interaction potential 3 points), a solvent model with an orthorhombic box was chosen. In the simulation, the OPLS 2005 force field was used [20]. To make models neutral, counter ions were introduced. To mimic physiological conditions, 0.15 m NaCl was added. The NPT ensemble with 300 K temperature and 1 atm pressure was chosen for the entire simulation. The models were relaxed before the simulation. The trajectories were saved for examination after every 100 ps, and the simulation's stability was verified by comparing the root mean square deviation (RMSD) values of protein and ligand over time.

## 3. Results

### 3.1. Protein-Ligand Docking

Molecular docking predicts the intermolecular framework and binding interactions between ligand molecules and proteins. Different docking approaches play a leading role in drug discovery. This study includes the protein-ligand docking and peptide-protein docking of twenty anti-inflammatory peptides counter to IFN-*γ*, IL-3, and TNF-alpha. The top three hit peptides from each analysis were selected on the basis of energy structure and interactions with active amino acids of the respective receptor protein (Table 1).

### 3.2. Interaction Analyses

Amongst twenty peptides as ligands, the peptide DEDTQAMMPFR showed the best interactions counter to IFN-*γ* and TNF-*α*. The peptide with *S*-score of -11.31 showed interactions with Lys34, Arg42, Gln46, and Tyr53 amino acids of the binding pocket of IFN-*γ* (Figure 1). The second peptide, QEPQESQQ with *S*-score of -10.98, exhibited interactions with Val22 and Glu39 residues of IFN-*γ* as a receptor protein (Figure S1). The third peptide FRDEHKK with *S*-score of -10.55 showed interactions with amino acids Val5, Glu39, and Tyr53 of IFN-*γ* (Figure S2). IFN-*γ* is a dimerized cytokine and known for its critical role in adaptive and innate immunity against variety of pathogens [21]. In addition to immunity response, it also activates a proinflammatory program in macrophages. The elevated level of IFN-*γ* has been observed in autoimmune complications including SLE [22].

The article "Identification of Peptides as Novel Inhibitors to Target IFN-γ, IL-3, and TNF-α in Systemic Lupus Erythematosus" was retracted in 2024. Reasons: signs of a paper mill; suspected computer-generated content; unreliable results or conclusions; concerns about the data.

For the IL-3, the peptide KHDRGDEF with *S*-score of -8.81 showed interactions with Cys16, Cys84, Pro86, and Leu87 amino acids of the binding pocket of IL-3 (Figure 2). The peptide FRDEHKK with *S*-score of -8.64 showed interactions with Asn15, Asp21, and Glu119 (Figure S3), and the peptide QEPQESQQ with *S*-score of -8.17 interacted with Pro83, Ala121, and Glu119 residues of IL-3 (Figure S4). Interleukin-3 is a multispecific hemopoietin, a glycoprotein cytokine that is synthesized by T cells in response to antigen. IL-3 has been involved in the proliferation and differentiation of many immune cells and both primitive multipotent and committed myeloid progenitors' cells [23, 24]. Elevated levels and increased IL-3-responsive progenitor cells have been reported in SLE patients [4].

The other receptor protein TNF-*α* is an inflammatory cytokine and important for resistance to cancer and infection. The dysregulation and elevation of this protein has been associated with many autoimmune disorders. In our study, the peptide DEDTQAMMPFR with *S*-score of -8.20 showed interactions with Arg32 and Leu142 amino acids of the binding pocket of TNF-*α* (Figure 3). Other peptides (i.e., FRDEHKK and QEPQESQQ) with *S*-scores of -7.32 and -7.25 interacted with Asp143, Pro20 and Glu23 (Figure S5), and Arg32 amino acids (Figure S6) in the binding pocket of TNF-*α*, respectively. TNF-*α* is a proinflammatory cytokine, belongs to the super family of tumor necrosis factor, and secreted by macrophages in a defense mechanism to protect from damage by inducing inflammation against pathogenic stimuli. The elevated level or mutation in TNF-*α* signaling leads towards deleterious consequences including many autoimmune disorders [25].

Collectively, with IFN-*γ*, IL-3, and TNF-*α*, many other cytokines and different factors have been studied to understand the autoimmunity events. Thus, there is an immediate need for the present age to understand the autoimmunity to control excessive inflammatory responses and balance cytokine signaling.

### 3.3. Peptide-Protein Docking

Peptide-protein interactions play a crucial role in a variety of regulatory and signaling pathways of the cell. The peptide-protein complex helps to open the key to elucidate important biological processes and to understand the underlying peptide-protein interactions. In this study, we used the top three ligands obtained from protein-ligand docking analysis for peptide-protein docking studies. The BLASTp was used to find suitable homologs and templates to build 3D structures of selected peptides in pdb format. Modeller 9.21 was employed for 3D structure predictions, and accurate models were selected on the basis of their DOPE values and GA341 scores. The HADDOCK server was used for docking of respective peptides counter to IFN-*γ*, IL-3, and TNF-*α* receptor proteins. Amongst selected peptides, only one peptide (i.e., DEDTQAMMPFR) with the HADDOCK score of −10.3 ± 2.5 kcal/mol showed binding with IFN-*γ* (Figure 4). The educational version of PyMOL was used to visualize and draw the predicted cluster of peptide protein. The remaining two peptides counter to IL-3 and TNF-*α* are not discussed here due to their poor HADDOCK scores and energy structures.

The article "Identification of Peptides as Novel Inhibitors to Target IFN-γ, IL-3, and TNF-α in Systemic Lupus Erythematosus" was retracted in 2024. Reasons: signs of a paper mill; suspected computer-generated content; unreliable results or conclusions; concerns about the data.

#### 3.3.1. MD Simulation

The evolution of RMSD values for the C-alpha atoms of protein-ligand complex over time has been shown in Figure 5(a). The plot showed that the complex reached stability at 10 ns. This was increase in RMSD of peptide at 50 ns. After that, for the length of the simulation, fluctuations in RMSD values for target remained within 1.5 Angstrom which is absolutely acceptable [26]. The ligand fit to protein RMSD values fluctuated within 1.5 Angstrom after they have been equilibrated. These findings indicate that the peptide stayed firmly connected to the receptor throughout the simulation period.

On the RMSF graphic (Figure 5(b)), peaks represented the portions of the protein that fluctuated the most during the simulation. Protein tails (both N- and C-terminal) typically changed more than any other part of the protein. Alpha helices and beta strands, for example, are usually stiffer than the unstructured section of the protein and fluctuate less than loop portions. According to MD trajectories, the residues with greater peaks belonged to loop areas or N and C-terminal zones (Figure S7). Low RMSF values of binding site residues indicated that ligand binding to the protein is stable.

Alpha-helices and beta-strands are monitored as secondary structure elements during the simulation (SSE). The graph above depicts the distribution of SSE by residue index across the protein structure. Throughout the simulation, the left graphic showed the SSE composition for each trajectory frame while the right plot monitors each residue's SSE assignment through time.

Protein interactions with the ligand can be detected throughout the simulation. These interactions were categorized and summarized by types (Figure S7). The four types of protein-ligand interactions (or “contacts”) include hydrogen bonds, hydrophobic interactions, ionic interactions, and water bridges. The “Simulation Interactions Diagram” panel in Maestro was used to study the subtypes of each interaction type. Over the course of the trajectory, the stacked bar charts were standardized: for example, a value of 0.7 indicated that the specific interaction was maintained for 70% of the simulation duration. Because some protein residues may make several interactions of the same subtype with the ligand, values above 1.0 are feasible. The majority of the significant ligand–protein interactions discovered by MD were hydrogen bonds and hydrophobic interactions (Figure 6). B:THR_27, D:GLY_75, and D:ASN_136 are the most important in terms of H-bond, and D:MET_25, D:PRO_77, and D:PRO_146 are the most important in terms of hydrophobic interactions.

The article "Identification of Peptides as Novel Inhibitors to Target IFN-γ, IL-3, and TNF-α in Systemic Lupus Erythematosus" was retracted in 2024. Reasons: signs of a paper mill; suspected computer-generated content; unreliable results or conclusions; concerns about the data.

A timeline has exhibited the interactions and contacts (H-bonds, hydrophobic, ionic and water bridges) as described above. In Figure 7, the top panel displayed the total number of specific connections the protein made with the ligand over the duration of the journey. The bottom panel of each trajectory frame showed which residues interacted with the ligand. Some residues made many particular connections with the ligand which has been indicated by a deeper shade of orange color according to the scale to the right of the plot.

Over the course of the trajectory, the stacked bar charts were standardized: for example, a value of 1.0 signified that the exact interaction was maintained for 100% of the simulation duration. Values exceeding 1.0 are possible because some protein residues may make several interactions of the same subtype with the ligand. The interactions of individual ligand atom with protein residues are showed in Figure 8. Interactions that last more than 30% of the simulation period in the selected trajectory (0.00 to 100.0 nsec) are shown.

The MMGBSA.py script from the Desmond module of the Schrodinger suite 2019-4 was used to perform the MM-GBSA analysis. Every frame was collected from each MD trajectory for binding free energy estimates of the receptor in combination with the peptide (Figure 9). Total energy was ranged from -996.226 to 5.056. The mean and median were -356.755 and -343.800, respectively, indicating good energy. Total binding free energy (kcal/mol) was calculated using the law of additivity in which individual energy modules such as coulombic, covalent, hydrogen bond, van der Waals, self-contact, lipophilic, solvation, and *π*–*π* stackings of the ligand and the protein were added together [27].

## 4. Discussion

Molecular docking is an elaborative approach to foresee the interactions between ligand and targeted amino acids in the binding pocket of the receptor protein [28]. Computational approaches including molecular docking help scientists to predict the binding capacities of different small molecules and peptides as drug candidates against different receptor proteins [29]. In the current study, we have used some plant- and animal-derived anti-inflammatory peptides ranging from 3 to 15 amino acid residues as ligands/peptides counter to proteins from different bacteria which are the leading cause of many autoimmune disorders.

The article "Identification of Peptides as Novel Inhibitors to Target IFN-γ, IL-3, and TNF-α in Systemic Lupus Erythematosus" was retracted in 2024. Reasons: signs of a paper mill; suspected computer-generated content; unreliable results or conclusions; concerns about the data.

The autoimmune disease SLE is a disorder of connective tissues with a wide range of clinical manifestations. The autoreactive B (bone marrow- or bursa-derived cells) and T cells (thymus cells) of adaptive and innate immunity play a leading role in the production of autoantibodies and lead towards autoimmune disorders including SLE [6]. Different factors such as IL-3, IL23, M-CSF, IFN-*α*, IFN-*γ*, and IL-6 have been reported in different studies to be involved in the production of autoantibodies but the main trigger for all these autoimmune complexities is still unknown [4, 30]. The elevated levels of proinflammatory cytokines and TNF-*α* have been reported in many studies as associated mainly with autoreactive B cells and T cells to produce autoantibodies [4, 6].

IFN-*γ* or type II interferon is a pleiotropic cytokine that coordinates with a diverse array of cellular immunity processes [31]. IFN-*γ* is a homodimer and formed by noncovalent interactions of 17 kDa polypeptide dimers and crucially known for early control of pathogen spreading. IFN-*γ* has been secreted mainly by CD4 T helper cells, CD8 cytotoxic T cells, and to a less extent by antigen-presenting cells (APCs) and natural killer cells [32]. The peripheral blood mononuclear cells (PBMCs) of SLE patients showed high level of IFN-*γ* transcript, and the T cells of SLE patients produce much more IFN-*γ* as compared to normal cells [33]. In the current study, strong interactions of three peptides (i.e., DEDTQAMMPFR, QEPQESQQ, and FRDEHKK) were found with the active amino acids present in the binding pocket of IFN-*γ* which could be used as potential inhibitors of IFN-*γ* to treat SLE.

IL-3 is a monomeric glycoprotein which is predominately produced by activated T cells in response to stimuli. It serves as a bridge between the immune system (T-lymphocytes) and the hemopoietic system that in response to foreign stimuli generates cellular elements for cellular defense [23]. The dysregulation of IL-3 has been associated with various autoimmune diseases including arthritis and SLE. In SLE patients, elevated IL-3 responsive progenitor cells have been observed in spleen, which show an association between IL-3 and autoreactive cells [4]. The molecular docking approach used in this study exhibited strong interactions of three peptides (i.e., KHDRGDEF, FRDEHKK, and QEPQESQQ) with the active amino acids present in the binding pocket of IL-3. These peptides could be potential inhibitors of IL-3.

The article "Identification of Peptides as Novel Inhibitors to Target IFN-γ, IL-3, and TNF-α in Systemic Lupus Erythematosus" was retracted in 2024. Reasons: signs of a paper mill; suspected computer-generated content; unreliable results or conclusions; concerns about the data.

TNF-*α* is a pleiotropic proinflammatory cytokine and contributes importantly to the development of B and T cells. TNF-*α* is a potent inflammatory mediator of chronic and acute inflammation and secreted by macrophages, T cells, and neutrophils [34]. The involvement of TNF-*α* in the pathogenesis of SLE has been observed in many clinical studies due to overexpression and elevated levels of TNF-*α* in SLE patients [35]. In current study, using molecular docking approach, three peptides (i.e., DEDTQAMMPFR, FRDEHKK, and QEPQESQQ) showed strong interactions with the active amino acids present in the binding pocket of TNF-*α* and could be used in the treatment of SLE.

The overexpression and elevated levels of interferons, interleukins, and tumor necrosis factor point towards the relationship of these factors to the pathogenesis of SLE and many other autoimmune disorders. The blockage of IFN-*γ*, IL-3, and TNF-*α* could be proved as an effective strategy to control the tissue and organ damage in SLE. In clinical trials, there are many ongoing therapies to control signaling pathways and targeted autoantibodies. Till now, many drugs have been approved and marketized such as rituximab, epratuzumab, abetimus, sodium, obinutuzumab, lulizumab pegol, abatacept, and blisibimod for the treatment of autoimmune disorders. The drug blisibimod is a fusion protein which is an antagonist of BAFF with little encouraging outcomes obtained after a phase III trial for the treatment of SLE [30]. In spite of many drugs and combinational therapies, these drugs have been associated with severe after effects; so, there is a need of such types of drugs with maximum potency and minimum side effects.

The proinflammatory cytokines, interleukins, and interferons make up the defense system of the cell and play a crucial role in generating different molecules in response to external pathogenic stimuli. Any mutation and overexpression of any of these molecules lead towards the production of autoantibodies against body's own cells. The peptides reported in this study could be used as potential drug candidates counter to IFN-*γ*, IL-3, and TNF-*α* as receptor proteins. Further elaborative study is still needed to explore much more potential of these anti-inflammatory peptides.

## 5. Conclusion

The docking analysis and *S*-scores of selected peptides have revealed the potential of selected peptides as drug candidates counter to inflammatory autoreactive proteins to control autoimmunity. In the current study, we used two types of docking analysis (protein-ligand and peptide-protein docking) to check the configuration and orientation of ligands/peptides counter to selected receptor proteins. In our first approach, the peptide DEDTQAMMPFR showed strong interactions with active amino acids of IFN-*γ* (*S*-score -11.31) and TNF-*α* (*S*-score 8.20) receptor proteins. The conformations showed the occupancy of the maximum binding pocket by ligand molecules. In our second approach (peptide-protein docking), the same peptide also showed strong bonding with the active amino acids of IFN-*γ* via HADDOCK server. The IFN-*γ*-DEDTQAMMPFR complex with HADDOCK score of −10.3 ± 2.5 kcal/mol showed strong interactions amongst active amino acid residues of both peptide and receptor protein. Further, the MD simulation analysis also confirmed that the peptide stayed firmly connected to the receptor throughout the simulation period (i.e., 120 nanoseconds). The results of the current study have explored the potential of peptides of plant and animal sources as drug molecules to control autoimmunity. The study could be proved as an initial step for further use of these peptides after some required modifications as drug candidates against autoimmune disorders.

The article "Identification of Peptides as Novel Inhibitors to Target IFN-γ, IL-3, and TNF-α in Systemic Lupus Erythematosus" was retracted in 2024. Reasons: signs of a paper mill; suspected computer-generated content; unreliable results or conclusions; concerns about the data.

## Figures and Tables

**Figure 1:** Binding interactions of peptide DEDTQAMMPFR with receptor IFN-*γ* revealed through protein-ligand approach. (a) Interactions of peptide with the receptor. The Gln46 and Tyr53 are polar amino acids and acting as sidechain acceptor and donor, respectively. Arg42 and Lys34 are basic amino acids and acting as sidechain donor and acceptor, respectively. (b) Binding patterns of peptide with the receptor protein.

**Figure 2:** Binding interactions of peptide KHDRGDEF with receptor IL-3 revealed through protein-ligand approach. (a) Interactions of peptide with the receptor. The Cys16 Cys84 are polar amino acids and acting as sidechain and backbone acceptors, respectively. Pro86 and Leu87 are greasy amino acids and acting as sidechain acceptor and backbone donor, respectively. (b) Binding patterns of peptide with the receptor protein.

**Figure 3:** Binding interactions of peptide DEDTQAMMPFR with receptor TNF-*α* revealed through protein-ligand approach. (a) Interactions of peptide with the receptor. Arg32 is a basic amino acid and acting as a sidechain donor while Leu142 is a greasy amino acid and acting as a backbone acceptor. (b) Binding patterns of peptide with the receptor protein.

**Figure 4:** Peptide-protein interactions between DEDTQAMMPFR and IFN-*γ*. The peptide DEDTQAMMPFR has been represented in yellow color with deep blue-colored interacting residues, and IFN-*γ* is shown in violet color with red interacting residues.

**Figure 5:** Root mean square deviation (RMSD) and residue wise root mean square fluctuation (RMSF). (a) RMSD of the C-alpha atoms of protein and ligand with time (receptor-peptide complex). The left *Y*-axis shows the variation of protein RMSD through time. The right *Y*-axis shows the variation of ligand RMSD through time. (b) RMSF of the protein.

The article "Identification of Peptides as Novel Inhibitors to Target IFN-γ, IL-3, and TNF-α in Systemic Lupus Erythematosus" was retracted in 2024. Reasons: signs of a paper mill; suspected computer-generated content; unreliable results or conclusions; concerns about the data.

**Figure 6:** Protein-ligand contact histogram (H-bonds, hydrophobic, ionic, water bridges).

**Figure 7:** A timeline representation of the interactions and contacts (H-bonds, hydrophobic, ionic, and water bridges).

**Figure 8:** Ligand atom interactions with the protein residues.

**Figure 9:** Estimation of binding free energy of the receptor in combination with the peptide using MM-GBSA.

**Table 1:** Top interactions of anti-inflammatory peptides with IFN-*γ*, IL-3, and TNF-alpha as receptor proteins.

Sr. No.	Peptide	Receptor	*S*-score	Interactions
1	DEDTQAMMPFR	IFN-*γ*	-11.30	Lys34, Arg42, Gln46, Tyr53
2	QEPQESQQ	IFN-*γ*	-10.98	Val22, Glu39
3	FRDEHKK	IFN-*γ*	-10.55	Val5, Glu39, Tyr53
4	KHDRGDEF	IL-3	-8.81	Cys16, Cys84, Pro86, Leu87
5	FRDEHKK	IL-3	-8.64	Asn15, Asp21, Glu119
6	QEPQESQQ	IL-3	-8.17	Pro83, Glu119, Ala121
7	DEDTQAMMPFR	TNF-*α*	-8.20	Arg32, Leu142
8	FRDEHKK	TNF-*α*	-7.32	Pro20, Glu23, Asp143
9	QEPQESQQ	TNF-*α*	-7.25	Arg32

## Data Availability

The data used to support the findings of this study are available from the corresponding author upon request.

## Supplementary Materials

Supplementary Materials Figure S1: interactions (a) and binding pattern (b) of QEPQESQQ peptide with IFN-*γ*. Figure S2: interactions (a) and binding pattern (b) of FRDEHKK peptide with IFN-*γ*. Figure S3: interactions (a) and binding pattern (b) of FRDEHKK peptide with IL-3. Figure S4: interactions (a) and binding pattern (b) of QEPQESQQ peptide with IL-3. Figure S5: interactions (a) and binding pattern (b) of FRDEHKK peptide with TNF-*α*. Figure S6: interactions (a) and binding pattern (b) of QEPQESQQ peptide with TNF-*α*. Figure S7: protein secondary structure element distribution by residue index throughout the protein structure (Supplementary Materials).
